The article "circSMARCA5 Promoted Osteosarcoma Cell Proliferation, Adhesion, Migration, and Invasion through a Competing Endogenous RNA Network" was retracted in 2024. Reasons: signs of a paper mill; suspected computer-generated content; unreliable results or conclusions; concerns about the data.

# circSMARCA5 Promoted Osteosarcoma Cell Proliferation, Adhesion, Migration, and Invasion through a Competing Endogenous RNA Network

**DOI:** 10.1155/2020/2539150

**Published:** 2020-09-27

**Authors:** Hepeng Zhang, Fanyu Meng, Shuaicheng Dong

**Affiliations:** ^1^The Health Center of Dongfu Township, North Forest District, Suihua City, China; ^2^Harbin Fourth Hospital, Harbin, China

## Abstract

Osteosarcoma (OS) is a widely common sort among bone cancer in children, and its overall survival ratio is low. The hidden mechanism of tumor genesis, progression, and metastasis regarding osteosarcoma needed to be further investigated. Emerging studies concentrated on exploring the functional roles of circular RNAs (circRNAs) in human cancers. The present study conducted a loss-of-function experiments to explore the circSMARCA5-induced influence on OS proliferation, cell cycle, and metastasis. Moreover, our manuscript unearthed the potential mechanisms of circSMARCA5 in regulating OS progression by in silico analysis. Our findings would provide new evidence to support that circSMARCA5 could be indicated as a biomarker for OS.

## 1. Introduction

Osteosarcoma occurs widely among bone cancer in children, and its overall survival proportion was unsatisfactory. The unknown role involved in tumor genesis, progression, and metastasis of osteosarcoma demanded further investigation. Over the past five years, emerging studies focused on exploring the functional roles of circular RNAs (circRNAs) in human cancers. circRNAs generated by a specific back-splicing mechanism belong to noncoding RNA clades. The mechanism of circRNAs in cancer progression involved sponging miRNAs, regulating parental gene expression, nuclear transportation, and translational machinery. For example, CDR1as could sponge miR-7 to promote its target gene expression [1]. circFoxo3 could interact with FAK and HIF-1*α* proteins to prevent their nuclear translocation [2]. Elaborating the duty of circRNAs will supply a new hint of defining diagnostic and therapeutic targets for osteosarcoma.

In previous studies, circRNAs had been found to play crucial roles in osteosarcoma [3]. circRNAs were involved in regulating multiple biological activities in osteosarcoma, comprising cell proliferation, migration, invasion, and chemoresistance. For instance, circPVT1 induced doxorubicin and cisplatin resistance of osteosarcoma [4]. circHIPK3 suppressed osteosarcoma proliferation, migration, and invasion [5]. However, circNASP was reported to induce osteosarcoma cell proliferation and invasion [6]. Very interestingly, circRNAs were found to be dysregulated which was correlated with the prognosis of osteosarcoma, indicating that circRNAs could be potential biomarkers for OS. Higher expression of hsa_circ_0007534 predicted poor prognosis of OS [7]. circSMARCA5 had been found to be upregulated in prostate cancer but downregulated in hepatocellular carcinoma, cervical cancer, and glioma. However, the molecular functions of circSMARCA5 in OS remained largely unclear.

Here, we executed a series of function experiments to uncover circSMARCA5-caused influence on OS proliferation, cell cycle, and metastasis. Moreover, the present study explored the potential mechanisms of circSMARCA5 regulating OS progression using in silico analysis. This study could provide new evidence to support that circSMARCA5 could be a biomarker for OS.

## 2. Material and Methods

### 2.1. Cell Culture and Transfection

HOS and MG-63 was derived from the Cell Bank of the Chinese Academy of Sciences (Shanghai, China) and then cultured in RPMI-1640 medium (Corning, USA) containing 10% FBS (HyClone, USA) under a 37°C incubator with 5% CO_2_.

As reported by Simon et al., we synthesized the sequence of circSMARCA5 siRNA from GenePharma (Shanghai, China). si-circSMARCA5 (5′-AAACAAAAGGGAGGCUUGUTT-3′) and scrambled siRNA (5′-UUCUCCGAACGUGUCACGUTT-3′) were separately transfected into cells by using the Lipofectamine 2000 reagent (Life, USA) as described in the manual.

### 2.2. Extraction and Quantification of RNA

Total RNA for RT-qPCR was harvested with the TRIeasy™ Total RNA Extraction Reagent (Yeasen, China). FastKing gDNA Dispelling RT SuperMix (TIANGEN, China) was used for reverse transcription (RT). An miR-29a-specific RT primer was supplied by GenePharma (Shanghai, China). For analysis of microRNA expression, qRT-PCR was performed using TransScript II Green One-Step qRT-PCR SuperMix (TransGen Biotech, China) on the LightCycler® 480. miR-29a expression level was obtained after, which was relative to U6. All PCR primers for mature miR-29a and U6 were ordered from HuaGene. The 2^-*ΔΔ*Ct^ method was applied to calculate relative miRNA expression. All the samples were tested three times [8].

### 2.3. Cell Adhesion Assay

Matrigel was formulated as a 0.04 *μ*g/*μ*l artificial basement membrane gel using the serum-free medium RPMI-1640. Matrigel 2 *μ*g per well was placed in a 96-well plate and then air-dried overnight in a superclean bench. 5000 cells in 100 *μ*l serum-free RPMI-1640 were inoculated in 96 wells and cultured for 2 hours; then, the cells that adhered to Matrigel were washed twice in PBS, fixed in methanol for 10 minutes, then dyed with DAPI, and observed under a fluorescent microscope (Olympus, Japan) to count the number of adherent cells. Each experiment was repeated three times.

### 2.4. Cell Invasion Assay

Transwell plates (8 mm pore size, 6.5 mm diameter; Corning Life Sciences, Lowell, MA) precoated with a Matrigel basement membrane matrix (1 mg/ml; BD Biosciences, Franklin Lakes, NJ) were applied to detect cell invasion. Briefly, HOS and MG-63 (5 × 10^4^ cells/well) were inoculated in the upper chamber of Transwell plates and incubated with RPMI-1640 containing 2% FBS. The bottom chamber of Transwell plates is full of RPMI-1640 supplemented with 10% FBS. At 24 hours postincubation, noninvasive cells in the upper chamber were discarded and invasive cells that had invaded through the Matrigel matrix membrane were dyed with crystal violet for 30 minutes. The inverted microscope was applied to count the amount of invading cells.

### 2.5. Statistical Analysis

All the data indicated as mean ± standard deviation (SD) are derived from more than three independent experiments. Based on the test conditions, statistical comparisons between standardized data sets were conducted using either the *t*-test or the Mann-Whitney *U* test. A *P* value not more than 0.05 indicates a significant difference, with a 95% confidence level.

## 3. Results

### 3.1. Knockdown of circSMARCA5 Expression in HOS and MG-63 Cells

circSMARCA5 expression was detected in osteosarcoma cells (HOS and MG-63) and osteoblast cells (OB3 cells). Our results showed that circSMARCA5 in HOS and MG-63 was greatly increased compared to that in OB3 cells (Figure 1(a)). Next, the RT-PCR assay was conducted to evaluate circSMARCA5 localization in OS cells. As shown in Figure 1(b), the present study found that circSMARCA5 was a cytoplasmic circRNA.

Then, the present study performed knockdown of the expression of circSMARCA5 using a specific siRNA reported by Simon et al., and our data revealed that circSMARCA5 RNA expression was hugely suppressed in both HOS and MG-63 cells after transfection (Figures 1(c) and 1(d)).

### 3.2. Cell Proliferation of OS Was Retarded by Reduced circSMARCA5

The CCK-8 assay was executed to detect circSMARCA5-induced influence on OS proliferation. Our data revealed that si-circSMARCA5-transfected HOS and MG-63 cells grew slower than those transfected with NC (Figures 2(a) and 2(b)).

Next, the flow cytometry method was applied to determine miR-135a-imposed effects on the OS cell cycle. As shown in Figures 2(c)–2(f), the results revealed that ablated circSMARCA5 impelled the ratio of the S and G2 phases but substantially decreased the ratio of the G1 phase in both HOS and MG-63 cells.

### 3.3. Downregulated circSMARCA5 Suppressed Cell Adhesion of HOS and MG-63

Cell adhesion was involved in regulating cancer metastasis processes. Thus, the present study conducted knockdown of circSMARCA5 and performed the cell adhesion assay in HOS and MG-63 cells. Both HOS and MG-63 cell adhesion in the circSMARCA5-knockdown group were largely decreased relative to those in NC groups (Figure 3).

### 3.4. The Knockdown of circSMARCA5 Inhibits HOS and MG-63 Cell Migration

The Transwell assays were performed to explore the effects of circSMARCA5 on the migration of OS cells. The results showed that migrating cells in the circSMARCA5-knockdown group were significantly reduced by 70% and 30% compared to both HOS and MG-63 cells in the control group (Figure 4). These results indicated that circSMARCA5 promoted HOS and MG-63 cell migration.

### 3.5. Knockdown of circSMARCA5 Suppressed HOS and MG-63 Cell Invasion

Our study also detected the effect of circSMARCA5 on OS invasion using Matrigel. The present study found that knockdown of circSMARCA5 suppressed cell invasion of HOS and MG-63 cells. The number of invading cells in the circSMARCA5-knockdown group was decreased by 70% and 50% compared to HOS and MG-63 cells in the control group (Figure 5).

### 3.6. Construction of circSMARCA5 Mediated the ceRNA Network in OS

To investigate the mechanisms of circSMARCA5 regulating OS proliferation and metastasis, the present study constructed a ceRNA network using the CircNet database (http://syslab5.nchu.edu.tw/CircNet/). As illustrated in Figure 6, there are a total of 5 miRNAs (miR-17-3p, miR-432-5p, miR-561-3p, miR-10b-3p, and miR-181c-3p) and 25 mRNAs (TXNRD2, OPTN, RBM5, TUBB4B, BPNT1, LRPPRC, CENPA, DNAJD6, ADAR, RNF103, HIPK3, RAB32, TBR1, ADSS, ADAMTS13, LILRB2, WDFY2, ARL4C, ARPP19, B3GALT5, ZNF730, STX6, RCAN2, CDKN1B, and LPCAT3).

## 4. Discussion

Previous studies had demonstrated that circRNAs played important roles in OS progression. circRNAs played as either oncogenes or tumor suppressors in OS. For example, circ_0000502 induced OS progression via sponging miR-1238 [9]. CDR1as induces OS tumor growth by sponging miR-7 [10]. circ_0001721 facilitates the progression of OS by way of sponging miR-569 and miR-599 [11]. However, circHIPK3 suppressed osteosarcoma proliferation, migration, and invasion [5]. Our manuscript validated circSMARCA5-mediated effects on the growth and metastasis of OS by a loss-of-function assay. Our manuscript found that circSMARCA5 level was upregulated in OS cells. Ablated circSMARCA5 level suppressed cell proliferation, cell cycle, and cell adhesion of OS. The Transwell assay revealed that decreased circSMARCA5 evidently inhibited OS cell migration and invasion. Taken together, the present study, for the first time, reported that circSMARCA5 played as an oncogene in OS.

SMARCA5 was involved in regulating nucleosome remodeling and transcription initiation. Several circRNA transcripts were transcribed from SMARCA5 genes, including hsa_circ_0001445, hsa_circ_0071043, hsa_circ_0071045, hsa_circ_0071044, hsa_circ_0071046, and hsa_circ_0071047. The present study focused on hsa_circ_0001445, which was found to be upregulated in epithelial to mesenchymal transition (EMT) progression. Simon et al. found QKI to regulate this transcript formation. Kong et al. found that overexpressed hsa_circ_0001445 was shown in prostate cancer, while hsa_circ_0001445 knockdown significantly repressed cell proliferation of PCa by inducing cell cycle arrest and apoptosis [12]. However, other groups showed that circSMARCA5 could also serve as a tumor suppressor. Li et al. found that hsa_circ_0001445 suppressed the proliferation and migration of hepatocellular carcinoma [13]. Meanwhile, circSMARCA5 was found to suppress the migration of glioblastoma through SRSF1/SRSF3/PTB [14], inhibiting cervical cancer cell proliferation, invasion, and migration through sponging microRNA-620 [15]. These reports, together with our findings, showed that circSMARCA5 might play different roles in different types of human cancers.

Considering that a single circRNA could sponge multiple miRNAs and a single miRNA could target multiple mRNAs, the present study constructed a circSMARCA5-mediated ceRNA network in OS using the CircNet database (http://syslab5.nchu.edu.tw/CircNet/). There are a total of 5 miRNAs (miR-17-3p, miR-432-5p, miR-561-3p, miR-10b-3p, and miR-181c-3p) and 25 mRNAs (TXNRD2, OPTN, RBM5, TUBB4B, BPNT1, LRPPRC, CENPA, DNAJD6, ADAR, RNF103, HIPK3, RAB32, TBR1, ADSS, ADAMTS13, LILRB2, WDFY2, ARL4C, ARPP19, B3GALT5, ZNF730, STX6, RCAN2, CDKN1B, LPCAT3). Among these genes, microRNA-432 was downregulated in OS and suppressed cell proliferation and invasion [16]. miR-181c was found to inhibit OS cell viability [17]. These reports supported our finding that circSMARCA5 played a carcinogenic part in OS.

However, there are some limitations in our manuscript. Firstly, though the results may have potential clinical applications, they still need clinical validation. Secondly, the selected miRNAs and mRNAs in the ceRNA network also need further validation.

## 5. Conclusion

Collectively, we for the first time showed that circSMARCA5 was an oncogene in OS by inducing cancer cell proliferation, adhesion, migration, and invasion. Mechanically, circSMARCA5 could sponge various OS growth- and metastasis-related miRNAs, including microRNA-432 and miR-181c. These results provided useful information to explore whether circSMARCA5 could serve as a diagnostic and therapeutic target for osteosarcoma.

## Figures and Tables

**Figure 1:** Knockdown of circSMARCA5 expression in HOS and MG-63 cells. (a) circSMARCA5 in HOS and MG-63 was apparently upregulated compared to that in OB3 cells. (b) circSMARCA5 was a cytoplasmic circRNA. (c, d) si-circSMARCA5 significantly suppressed circSMARCA5 expression in both HOS and MG-63 cells. ^∗^*P* < 0.05.

**Figure 2:** Knockdown of circSMARCA5 retarded cell proliferation of OS. (a, b) The knockdown of circSMARCA5 hindered cell proliferation of HOS and MG-63. (c–f) The knockdown of circSMARCA5 heightened the proportion of the S and G2 phases but substantially decreased the proportion of the G1 phase in both HOS and MG-63 cells. ^∗∗∗^*P* < 0.001.

**Figure 3:** Knockdown of circSMARCA5 suppressed HOS and MG-63 cell adhesion. (a–d) The knockdown of circSMARCA5 significantly suppressed the adhesion of both the HOS (a, b) and MG-63 (c, d) cells. ^∗^*P* < 0.05.

**Figure 4:** Knockdown of circSMARCA5 suppressed HOS and MG-63 cell migration. (a–d) The knockdown of circSMARCA5 significantly suppressed the migration of both the HOS (a, b) and MG-63 (c, d) cells. ^∗^*P* < 0.05, ^∗∗∗^*P* < 0.001.

**Figure 5:** Knockdown of circSMARCA5 suppressed HOS and MG-63 cell invasion. (a, d) The knockdown of circSMARCA5 significantly suppressed the invasion of both the HOS (a, b) and MG-63 (c, d) cells. ^∗^*P* < 0.05, ^∗∗∗^*P* < 0.001.

**Figure 6:** circSMARCA5 mediated the ceRNA network in osteosarcoma. There are a total of 5 miRNAs (miR-17-3p, miR-432-5p, miR-561-3p, miR-10b-3p, and miR-181c-3p) and 25 mRNAs (TXNRD2, OPTN, RBM5, TUBB4B, BPNT1, LRPPRC, CENPA, DNAJD6, ADAR, RNF103, HIPK3, RAB32, TBR1, ADSS, ADAMTS13, LILRB2, WDFY2, ARL4C, ARPP19, B3GALT5, ZNF730, STX6, RCAN2, CDKN1B, LPCAT3).

## Data Availability

All raw data can be made available upon request.

## References

[1] Yang W., Yang X., Wang X. (2019). Silencing CDR1as enhances the sensitivity of breast cancer cells to drug resistance by acting as a miR-7 sponge to down-regulate REG*γ*. *Journal of Cellular and Molecular Medicine*.

[2] Du W. W., Yang W., Chen Y. (2016). Foxo3 circular RNA promotes cardiac senescence by modulating multiple factors associated with stress and senescence responses. *European Heart Journal*.

[3] Soghli N., Qujeq D., Yousefi T., Soghli N. (2020). The regulatory functions of circular RNAs in osteosarcoma. *Genomics*.

[4] Kun-Peng Z., Xiao-Long M., Chun-Lin Z. (2018). Overexpressed circPVT1, a potential new circular RNA biomarker, contributes to doxorubicin and cisplatin resistance of osteosarcoma cells by regulating ABCB1. *International Journal of Biological Sciences*.

[5] Xiao-Long M., Kun-Peng Z., Chun-Lin Z. (2018). Circular RNA circ_HIPK3 is down-regulated and suppresses cell proliferation, migration and invasion in osteosarcoma. *Journal of Cancer*.

[6] Huang L., Chen M., Pan J., Yu W. (2018). Circular RNA circNASP modulates the malignant behaviors in osteosarcoma via miR-1253/FOXF1 pathway. *Biochemical and Biophysical Research Communications*.

[7] Li B., Li X. (2018). Overexpression of hsa_circ_0007534 predicts unfavorable prognosis for osteosarcoma and regulates cell growth and apoptosis by affecting AKT/GSK-3*β* signaling pathway. *Biomedicine & Pharmacotherapy*.

[8] Gu C., Huang Z., Chen X. (2020). TEAD4 promotes tumor development in patients with lung adenocarcinoma via ERK signaling pathway. *Biochimica et Biophysica Acta - Molecular Basis of Disease*.

[9] Qi H., Sun Y., Jiang Y., Li X. (2018). Upregulation of circular RNA circ_0000502 predicts unfavorable prognosis in osteosarcoma and facilitates cell progression via sponging miR-1238. *Journal of Cellular Biochemistry*.

[10] Xu B., Yang T., Wang Z., Zhang Y., Liu S., Shen M. (2018). CircRNA CDR1as/miR-7 signals promote tumor growth of osteosarcoma with a potential therapeutic and diagnostic value. *Cancer Management and Research*.

[11] Li L., Guo L., Yin G., Yu G., Zhao Y., Pan Y. (2019). Upregulation of circular RNA circ_0001721 predicts unfavorable prognosis in osteosarcoma and facilitates cell progression via sponging miR-569 and miR-599. *Biomedicine & Pharmacotherapy*.

[12] Kong Z., Wan X., Zhang Y. (2017). Androgen-responsive circular RNA circSMARCA5 is up-regulated and promotes cell proliferation in prostate cancer. *Biochemical and Biophysical Research Communications*.

[13] Li Z., Zhou Y., Yang G. (2019). Using circular RNA SMARCA5 as a potential novel biomarker for hepatocellular carcinoma. *Clinica Chimica Acta*.

[14] Barbagallo D., Caponnetto A., Cirnigliaro M. (2018). CircSMARCA5 inhibits migration of glioblastoma multiforme cells by regulating a molecular axis involving splicing factors SRSF1/SRSF3/PTB. *International Journal of Molecular Sciences*.

[15] Tian J. D. C., Liang L. (2018). Involvement of circular RNA SMARCA5/microRNA-620 axis in the regulation of cervical cancer cell proliferation, invasion and migration. *European Review for Medical and Pharmacological Sciences*.

[16] Lv D., Zhen Z., Huang D. (2019). MicroRNA-432 is downregulated in osteosarcoma and inhibits cell proliferation and invasion by directly targeting metastasis-associated in colon cancer-1. *Experimental and Therapeutic Medicine*.

[17] Fu Y., Tang Y., Wang J., Guo Z. (2019). MicroRNA-181c suppresses the biological progression of osteosarcoma via targeting SMAD7 and regulating transforming growth factor-*β* (TGF-*β*) signaling pathway. *Medical Science Monitor*.

